# Investigation of Effectiveness of Shuffled Frog-Leaping Optimizer in Training a Convolution Neural Network

**DOI:** 10.1155/2022/4703682

**Published:** 2022-03-23

**Authors:** Soroush Baseri Saadi, Nazanin Tataei Sarshar, Soroush Sadeghi, Ramin Ranjbarzadeh, Mersedeh Kooshki Forooshani, Malika Bendechache

**Affiliations:** ^1^Faculty of Medicine, Catholic University of Leuven (KU Leuven), Leuven, Belgium; ^2^Department of Engineering, Islamic Azad University, Tehran North Branch, Tehran, Iran; ^3^School of Electrical and Computer Engineering, University of Tehran, Tehran, Iran; ^4^School of Computing, Faculty of Engineering and Computing, Dublin City University, Dublin, Ireland; ^5^Department of Electronics and Telecommunications, Polytechnic University, Turin, Italy

## Abstract

One of the leading algorithms and architectures in deep learning is Convolution Neural Network (CNN). It represents a unique method for image processing, object detection, and classification. CNN has shown to be an efficient approach in the machine learning and computer vision fields. CNN is composed of several filters accompanied by nonlinear functions and pooling layers. It enforces limitations on the weights and interconnections of the neural network to create a good structure for processing spatial and temporal distributed data. A CNN can restrain the numbering of free parameters of the network through its weight-sharing property. However, the training of CNNs is a challenging approach. Some optimization techniques have been recently employed to optimize CNN's weight and biases such as Ant Colony Optimization, Genetic, Harmony Search, and Simulated Annealing. This paper employs the well-known nature-inspired algorithm called Shuffled Frog-Leaping Algorithm (SFLA) for training a classical CNN structure (LeNet-5), which has not been experienced before. The training method is investigated by employing four different datasets. To verify the study, the results are compared with some of the most famous evolutionary trainers: Whale Optimization Algorithm (WO), Bacteria Swarm Foraging Optimization (BFSO), and Ant Colony Optimization (ACO). The outcomes demonstrate that the SFL technique considerably improves the performance of the original LeNet-5 although using this algorithm slightly increases the training computation time. The results also demonstrate that the suggested algorithm presents high accuracy in classification and approximation in its mechanism.

## 1. Introduction

Currently, Deep Learning (DL) is the base for many cutting-edge artificial intelligence (AI) applications [1–3]. DL can learn features at a high-level state with more complexity and abstraction than shallower neural networks. It presents hierarchical features providing various methods, taking for instance, probabilistic models, and supervised and unsupervised methods [4, 5]. The most notorious feature of DL is its ability in reducing computer hardware and software manipulation, making advancements in computational capabilities, machine learning, and signal processing. Furthermore, it is proved to be a highly applicable solution in objects recognition [6–8], speech recognition [9–12], SAR image processing [13–16], and a highly viable method in medical image processing for the detection of potential drug molecules activities [17, 18], liver and lung tumor segmentation [19, 20].

DL principle can be employed for the design of a variety of neural networks, among which Deep Neural Network (DNN), Recurrent Neural Network (RNN), and Convolution Neural Network (CNN) are the most popular. There are also generative and hybrid models of DL. For the former, some examples are Deep Belief Network (DBN) and Boltzmann Machine (DBM), and for the latter referring to a combination of discriminative and generative models, a well-known example is pretrained deep CNN using DBN. Between the various models of DL, the focus of this study is on CNN [4, 21].

DL has a great ability for resolving learning problems. However, this method is challenging to be trained for producing the optimal results. A CNN model learns many patterns through many weights and biases inside the convolutional layers. These weights and biases obtain their best possible values through a learning process with a large number of data. Actually, in a CNN model, the number of the training samples plays a crucial role in the obtaining best possible solution [22–24]. To achieve this goal, many optimization methods have been proposed for manipulating the value of these weights and biases. The most well-known algorithms are Adaptive Gradient methods. Basically, these methods modify the learning rate by a backpropagation strategy. These approaches reduce the learning rate if the gradient of parameters is large or vice versa. Stochastic gradient descent (SGD) is the most preferred technique among adaptive gradient methods [25]. Nevertheless, they proved to have poor performance especially when the network is large like CNN since the learning rate needs to be manually tuned in SGD. This significantly increases the training time for large-scale datasets [26, 27]. To overcome this obstacle and improve the efficiency of adaptive, new variants of adaptive gradient methods are proposed such as Nostalgic Adam [28], which place bigger weights on the past gradient compared to the recent gradient, or YOGI [29], which increases in effective learning rate to achieve better convergence. However, they have not gained popularity for image processing applications with CNN, which gives rise to the use of Metaheuristic algorithms as alternatives.

Recently, metaheuristic methods have been employed to resolve complex problems such as scheduling [30] and detection problems [31]. The performance of metaheuristic algorithms in solving efficiently these problems makes them a good alternative to train neural networks with large parameters as they are simple to use, are independent form gradient, and avoid local optima [32, 33]. Metaheuristic algorithms could prove to be highly efficient in optimizing CNN parameters with large image datasets specifically in the field of image analysis. In a study carried out by Zhang et al. [34], a metaheuristic optimizer is employed to pretrain the CNN for the classification of skin cancer images. To achieve this goal, the Whale Optimization Algorithm (WOA), one of the subgroups of metaheuristic methods, was applied to reduce the error rate during the learning process. Their WOA method considers half value precision as the cost function during skin cancer validation steps that contains the simplified measured error between the output of the system and the reference. The results of this study demonstrated the accuracy prominence of this algorithm compared to the other popular classification methods used in this study. In another study performed by da Silva et al. [35], the hyperparameters of a convolutional neural network were trained with Particle Swarm Optimization (PSO), another subgroup of metaheuristic algorithm, for the classification of lung cancers (classify nodule candidates, benign or malignant tumors, into nonnodules and nodules). They used two preprocessing steps including (1) employing each CT slice as a separate sample and (2) resizing of all the samples into 28 × 28. The PSO method optimizes the size of trainable filters, number of batches in the training, type of pooling, number of neurons in the hidden layer, and number of kernels in the convolutional layers. Although, in this study, a large dataset of CT images was used, PSO demonstrated the accuracy of 97.62%, sensitivity of 92.20%, and specificity of 98.64%. Hoseini et al. [36] proposed an AdaptAhead optimization technique to learn a Deep CNN with robust architecture in relation to the high volume data. They utilized several MR images of BRATS 2015 and BRATS 2016 data sets to validate the proposed method. Their model fails to utilize the technique of Nesterov and the adaptive learning rate in computing the gradient leading to failure to reach the optimal convergence point.

Metaheuristic algorithms can be categorized into the following subgroups [37–39]:

- Swarm based methods act based on animal social behavior like PSO [40, 41], WOA [42]
- Evolutionary methods act based on a natural evolutionary process like Genetic algorithm (GA) [43]
- Biological based optimizers like Satin Bowerbird Optimizer (SBO) [44]
- Human-based algorithms inspired from human behavior such as Life Choice Based Optimizer [45]
- System-based algorithms inspired by natural ecosystems such as Artificial Ecosystem-based Optimizer (AEO) [46]
- Physics-based methods that mimic the physical phenomenon in nature like Equilibrium optimizer [47] and Simulated Annealing [48]

In this paper, to overcome the problem of overfitting and convergence, we optimize the values of weight and biases of a LeNet-5 by an optimization algorithm. From the various types of metaheuristic algorithms, we used the Shuffled frog-leaping algorithm (SFLA) to optimize the performance of the LeNet-5 CNN [49]. This is conducted by changing the values of weight and biases inside the model to reach a high accuracy of the model. This optimizer belongs to the Swarm-based algorithms of metaheuristic algorithms inspired by the natural behavior of frogs in searching for food. The reason for using this optimizer is that, at the time of working on this research work, based on our knowledge, there is no research to employ SFLA in training CNN and to make a good comparison with other optimizers to show the ability of this optimizer for image classification. Moreover, in order to verify our results, we applied the other well-known optimizers WOA, Ant Colony Optimizer (ACO), and Bacteria Swarm Foraging Optimization (BFSO) for comparison.

This paper is organized as follows: Section 1 is an introduction, Section 2 presents a literature review of convolution neural networks, Section 3 explains the SFL Algorithm mechanism, Section 4 describes the design of proposed methods, Section 5 presents the result and discussion of the experiment, and lastly, Section 6 is the conclusion.

## 2. Convolutional Neural Network

Neural networks or artificial neural networks are computing systems that have been inspired by the human brain. In other words, these networks mimic the biological functions that are transmitted the signal to other neurons such as synapses in a biological brain [11, 50–52]. A neural network contains mathematical functions, which compute the weighted sum of multiple inputs, output, and activation functions. Specifically, these functions are layers of interconnected nodes, which are known as artificial neurons. The convolutional neural network is one of the various classes of neural networks, which is often applied to analyze and process the vision dataset. Nowadays, a CNN model has a critical role since fast growth in deep learning and artificial intelligence. It is necessary to mention that deep learning is a neural network that is composed of more than three layers and, as well as CNN, is used multiple layers, such as convolution, pooling, and fully connected layers to learn features and detect patterns of image [4, 53–55].

The convolutional layer is a critical component of CNN that uses the information of adjacent pixels as a linear operation to extract features. Each location of the tensor is calculated through an element-wise product between input tensor, which is an array of numbers and kernel or filter, while its output is summed up in order to obtain a single value in the corresponding location of output tensor, which is known as a feature map. Several various kernels should be applied to represent a different characteristic of the input tensor in order to achieve variant feature extractors such as a horizontal edge detector or a vertical edge detector [4, 56]. The convolution operation reduces the size of the feature maps in comparison to the input tensor. Typically, the padding technique should be used to increase the dimension of the image and lose less information by adding zeros around the image. The stride is considered as a distance between two kernels in convolution operation, that is, commonly one, while sometimes usage of the values more than one is to obtain downsampling of feature map for a specified purpose [57, 58].

A pooling layer provides alternative and more robust downsampling, as well as avoiding overfitting and a lot of computation by representing abstracted feature maps. This layer is operated on each feature map independently to make a new set of the same number of pooled feature maps and reduce the number of subsequent learnable parameters. Specifically, filter size, stride, and padding are also applied as hyperparameters in pooling operations. There are two common functions in pooling operation, average pooling, which is computed average value for each patch of the feature map, and max pooling, which is calculated the maximum value. In all cases, polling supports that the value of pooled features is remained almost invariant by translating the small amount of input [4, 59, 60].

The linear output of convolution operation is passed through nonlinear activation function, which is considered as a fundamental component in order to learn the complex patterns and the ability to add nonlinearity into the network. There are various types of activation functions such as sigmoid or hyperbolic tangent function, which are taken into account as smooth nonlinear functions and rectified linear unit (ReLU) function, which is recently the most widely used activation function. This is due to the fact that sigmoid and tanh activation functions are commonly saturated and really sensitive to modify around their mid-point of their input [55, 61].

Typically, the output of the final convolution and pooling layer is transformed to a one-dimension array of numbers, which is known as flattening. The output of flattening is considered as the input of one or more fully connected layers, in which every neuron in one layer is connected to every neuron in the other layer. In other words, the nonlinear combination of high-level features, which is the output of the convolution layer, is learned by a fully connected layer in order to map the final output of the network such as the probability of each class in the classification task [4, 62]. It is important to mention that each fully connected layer is followed by an activation function such as ReLU except the last nonlinear function that is usually different from the others. The last activation function, which is applied in the classification task, is Softmax to obtain a probability of the input being in the specified class [58, 63, 64].

The cost function is another essential component in Neural Networks. Actually, cost and loss functions are synonymous; the only difference is that the single training batch uses the loss function, while the cost function is referred to apply the loss function over the entire training set. The loss function is evaluated by the compatibility between the predicted value and the ground truth label, in which the higher output of loss means the incapable performance of the model. Another hyperparameter that is required for assigning is selecting an appropriate loss function with respect to the performed task. Since the problem is an optimization problem, Gradient descent is usually applied as an optimization algorithm to minimize the loss function [4, 65, 66].

The type of CNN employed in this study is LeNet-5, which is one of the earliest CNN models [49] (Figure 1). It is a classical CNN developed originally for recognizing characters. The architecture of LeNet-5 is composed of seven layers, in which, except the input layer, the rest can be trained (weights). As shown in the Figure 1, the LeNet-5 network possesses three convolutional layers C1, C3, and C5 among its processing layers. These convolutional layers are composed of two pooling layers S2 and S4, and the output layer is F6. The arrangement of convolutional layers and subsampling layers is in the form of plans and form feature maps. Each neuron in convolutional layers is linked locally to the local receptive field in the previous layer. Neurons that have the same feature maps obtain data from different local receptive fields. This process continues until the entire input plane is skimmed, and similar weights are employed together. Feature maps are spatially downsampled in the subsampling layer, and their size is reduced by a factor of 2. There is a similar kernel size of 5 × 5 for the three convolution layers C1, C3, and C5. However, the numbers of feature maps and parameters for each layer are different from each other (Table 1). The last convolution layer C5 is fully connected to the S4, and it has the feature maps size of 1 × 1. F6 is the last layer that performs the classification task. This layer is composed of 84 units and fully connected to the last convolutional layer C5.

Essentially, convolution layers are connected to several feature maps, kernels, and correlated to the prior layers. Each extracted feature matrix (feature map) is generated as a consequence of a sum of convolution from extracted feature matrices of the earlier layer, their corresponding mask (kernel), and a linear filter. Moreover, a bias value is summed to the extracted feature matrix and subsequently; it is applied to a nonlinear function. The tanh function is employed for this purpose. The *k*th feature map *M*_*ij*_^*k*^ with the weights *W*^*k* ^ and *b*_*k*_  is achieved by applying the tanh function as follows:

(1) $$\begin{array}{c} M_{ij}^{k}=\text{tanh}\left({\left(\;W^{k}\times x\right)}_{ij}+b_{k}\right). \end{array}$$

Through a subsampling layer, the size of each extracted feature matrix is reduced in relation to one of the extracted feature matrices of the former layer. This pooling strategy decreases the resolution of the extracted feature matrix. The pooling layers summarize the features present in an area of the feature map created by convolution layers. Also, a pooling layer diminishes the number of parameters for learning and the amount of computation performed in the network.

The classification task is carried out through the classification layer. This layer is placed after all the convolution and subsampling layers. In the classification layer, the output of each neuron is given to a single class label, and in the case of Oxford17, Oxford 102, Caltech/UCSD birds, and Caltech 101 airplanes dataset, this layer is composed often neurons corresponding to their labels.

## 3. Shuffled Frog-Leaping Optimizer

Shuffled Frog-Leaping Algorithm (SFLA) is a memetic metaheuristic approach that is employed to find a global solution through an informed heuristic search by employing a heuristic function [67]. This algorithm is a population-based technique that is occasioned by natural memetic. The term memetic is coming from “meme” considered as the unit of cultural evolution. Theoretically, the SFLA is similar to the particle swarm optimization (PSO). However, the values of weights and biases can be exchanged among local searches through a shuffling technique, thereby obtaining global optimum. The genuine aims of genes and memes are different from each other since they apply different mechanisms for data distribution from one population member to another [68, 69]. Gene's transmission is only possible from parents to offspring and only occurs between generations. However, memes can be transmitted between any two individuals, and instead of waiting for a full generation of genes to be replicated, it can cooperate with other memes immediately once an improved idea is found. Moreover, the replication of the genes is limited to the slight number of offspring that can belong to a single parent. On the other hand, a meme can be taken over by an unlimited number of individuals [70].

SFL algorithm is a population-based approach composed of frogs of the same attributes. Each frog can be considered as a solution. The total population of frogs is divided into numerous subgroups known as memeplexes. Diverse subgroups can be appreciated as dissimilar frog memes. Each memeplex is responsible for a limited exploration. At each memeplex, other frogs might affect the behavior of each frog, and the evolution will take place through the process of memetic evolution [70, 71]. After a number of memetic evolution periods, the memeplexes are forced to join together leading to the generation of novel memeplexes through a shuffling method. Shuffling will completely make unbiased the cultural evolution in the direction of any specific interest. The stopping criteria are satisfied once the local search and the shuffling procedure alternate [68]. The flowchart of SFLA is shown in Figure 2. The different steps are described as follows [67, 72, 73]:

(1) The algorithm contains a population “*p*” of the potential number of solutions, controlled by a set of virtual frogs (*n*).
(2) The population is split into subsets denoted as memeplexes (*m*). The memeplexes can be considered as a set of parallel frog cultures trying to achieve some goals.
(3) Frog *i* is shown by *X*_i_ = (*X*_*i*1_, *X*_*i*2_,…, *X*_*is*_) in which *S* indicates the number of variables.
(4) Within each memeplex, each frog culture searches the space in different directions and exchanges ideas independently. The frogs with best and worst fitness are denoted as *X*_b_ and *X*_*w*_.
(5) Frog with global best fitness is identified as *X*_*g*_.
(6) The frog with the worst fitness is modified based on the following equation:
  (2) $$\begin{array}{c} D_{i}=\text{rand}\left(X_{b}-X_{w}\right),\\ X_{\text{new}w}=X_{\text{old}W}+D_{i}\;\left(-D_{\text{max}}\leq D_{i}\leq D_{\max}\right), \end{array}$$

In which the rand function generates an arbitrary number between the range [0, 1], *D*_*i*_ is the size of the leaping step of the frog_*i*_ and *D*_max_ is the maximum value permitted to adjust frog position. If the value of fitness *X*_*w*_ is better than the current value of *X*_*w*_, it will be accepted. If the fitness value is not modified, then the calculation is repeated by replacing *X*_*b*_ with *X*_*g*_. If there is no potential for enhancement, a novel *X*_*w*_ will be created arbitrarily. This shuffling process and the local search continue until defined convergence criteria provide satisfactory results [68, 70, 71].

## 4. Design of Proposed Method

Problem representation is the foremost step in training a CNN employing metaheuristics algorithms. To train a CNN, the problem should be formulated in a suitable way for metaheuristics. The most important variables to training this type of network are weights and biases. In the trainer, the best biases and weights values are found to provide the highest classification, approximation, and prediction accuracy for the network. Thus, biases and weights are trainable variables. It means by changing the values of biases and weights of all neurons the output results of the network can be varied. So, controlling the process of applying new weights and biases by an optimizer approach leads to reaching higher accuracy. As the SFL procedure takes the variables in the format of a vector, the variables of a CNN denoted for this technique are as follows:

(3) $$\begin{array}{c} \overset{⟶}{V}=\left\{\overset{⟶}{W},\;\overset{⟶}{\theta }\right\}=\left\{W_{1,1},\;W_{1,2},\ldots ,\;W_{n,n},h,\theta_{1},\theta_{2},\ldots ,\theta_{h}\right\}. \end{array}$$

In which *n* is the size of the input, *W*_*ij*_  denotes the connection weight between layers *i*th and *j*th, and *θ*_*j*_ is the bias (threshold) of the *j*th hidden node.

Once the variables are defined, defining the objective function for the SFL technique is the next goal. Mean Square Error (MSE) is a common metric for the evaluation of networks. Once a set of training samples are given to the CNN, this equation measures the difference between the obtained output values and the desirable values through the following equation:

(4) $$\begin{array}{c} \text{MSE}=\sum_{i=2}^{m}\left(o_{i}^{k}-d_{i}^{k}\right), \end{array}$$

where *m* indicates the output numbers, the preferred output of the *i*th input unit when the *k*th training data samples are utilized is denoted by *d*_*i*_^*k*^, and the actual output of the *i*th input unit when the k*th* training data appear in the input is *o*_*i*_^*k*^.

To design an effective CNN, the network should be adapted to the whole set of training samples. As a result, CNN performance is assessed according to the average of MSE with respect to the training samples as the following equation:

(5) $$\begin{array}{c} \bar{\text{MSE}}=\sum_{k=1}^{s}\frac{\sum_{i=1}^{m}{\left(o_{i}^{k}-d_{i}^{k}\right)}^{2}²}{s},\\ \text{Minimize:}F\left(\overset{⟶}{v}\right)=\bar{\text{MSE}}. \end{array}$$

As, at each iteration, the weights and biases move towards having the best CNN, the probability of an improved CNN increases gradually. However, due to stochastic nature of SFL algorithm, there is no guarantee that the optimal CNN is obtained. On the other hand, with sufficient number of iteration, the SFL algorithm finally reaches to a solution that works more efficient than random preliminary solutions. The following section assesses the advantages of the SFL algorithm in training a CNN practically.

## 5. Experimental Results and Discussion

In this part, the suggested SFL-based CNN is investigated by employing four standard classification datasets from [74–77], OxFord Flowers 17 (Figure 3(a)), OxFord Flowers 102 (Figure 3(b)), Caltech/UCSD Birds (Figure 3(c)), and Caltech 101 Airplanes (Figure 3(d)). The specifications of the datasets are presented in Table 2.

The classification datasets were intentionally selected with the diverse test/training data and difficulty levels to efficiently evaluate the performance of our SFL-based CNN. We employed a Hewlett-Packard (hp) computer with the processor of Intel (R) Core (TM) i7-6500U CPU @ 2.50 GHz 2.60 GHz, installed memory (RAM) of 8.00 GB, System type of 64-bit Operating System, and Windows 10 Home. For data processing, we used MATLAB and Statistics Toolbox Release 2019a. The SFL assumptions and other techniques are shown in Table 3. The accuracy of classification for each dataset using different optimization algorithms is demonstrated in Figure 4. It is considered that the optimization method begins by creating random biases and weights in the range of [−10, 10] for all four datasets.

To generate the results, the datasets are solved 50 times by applying each technique. As illustrated in Figure 4, after the last iteration, the error of classification for all the datasets employing different optimizers decreases to approximately less than 10%, in which the SFL algorithm appears to be the most efficient optimizer. The average (AVE) and standard deviation (STD) shown in Tables 4–7 are actually the best MSEs obtained in the last iteration. Clearly, the lowest average and standard deviation of MSE in the final iteration illustrate the best result. The statistical outcomes are shown in the form of AVE ± STD. It should be noted that the best rates of classification attained by each method during 50 iterations are reported as another metric of comparison. Statically analysis of the results shows that training CNN with SFL algorithm provides the best accuracy of classification in all the mentioned datasets, as well as superior local optima avoidance, which is the reason for the improved MSE. Moreover, the results of this study demonstrate that, unlike other swarm-based algorithms, SFL algorithm has a better performance since it does not have a mechanism for substantial sudden movements to search the space. It is also demonstrated that ACO and WO optimizers reach a minimum time for training the model in comparison of BFSO and SFL methods. Also, the SFL method takes more time than ACO and WO approaches, but it obtains higher classification rates and minimum MSE scores.

## 6. Conclusion

This study presented Shuffled Frog-Leaping Algorithm (SFLA) as one model of metaheuristic algorithms to optimize one type of Convolutional Neural Network. At first, the training problem of a CNN was formulated for the SFL technique. This method was then applied to define the optimum values for biases and weights. Theoretically, the SFLA is similar to the particle swarm optimization (PSO). However, the values of weights and biases can be exchanged among local searches through a shuffling technique, thereby obtaining global optimum. The proposed SFLA was employed to train four standard classification datasets (OxFord Flowers 17, OxFord Flowers 102, Caltech/UCSD Birds, and Caltech 101 Airplanes). To verify the performance of SFLA, the results were compared to three other stochastic optimization trainers: WO, BFSO, and ACO. The resulting outcomes demonstrated that the suggested technique can effectively train the CNN. It improves the probability of finding optimal values for biases and weights for CNNs. Our optimization strategy can obtain noticeable accuracy for classifying objects in four standard classification datasets.

For future study, finding the proper parameters for SFL algorithm needs to be investigated. Moreover, by exploring the optimal values for number of batches in the training, type of pooling, number of neurons in the hidden layer, and number of kernels in the convolutional layers, we can obtain more noticeable results. Further optimal tuning of this method is worth further research using different datasets such as CKP and facial expression datasets, as well as ImageNet and ORI.

## Figures and Tables

**Figure 1:** Illustration of LeNet-5 architecture, a convolution neural network. Each plan in the network indicates a feature map [48].

**Figure 2:** Flowchart of SFL algorithm.

**Figure 3:** Datasets sample pictures. (a) OxFord flowers 17. (b) OxFord flowers 102. (c) Caltech/UCSD birds. (d) Caltech 101 airplanes.

**Figure 4:** Error of classification using different datasets and optimization algorithms for LeNet-5. (a) OxFord flowers 17. (b) OxFord flowers 102. (c) Caltech/UCSD birds. (d) Caltech 101 airplanes.

**Table 1:** Properties of the layers of the LeNet-5 [48].

Layer	Size	Num. of feature maps	Num. of parameters	Num. of connections
Input	32 × 32	…	…	…
C1	28 × 28	6	156	122304
S2	14 × 14	6	12	5880
C3	10 × 10	16	1516	151600
S4	5 × 5	16	32	2000
C5	1 × 1	120	…	48120
F6	1 × 1	84	10164	…

**Table 2:** Dataset specifications.

Dataset	Number of categories	Number of images per category	Training sample numbers	Test sample numbers
OxFord flowers 17	17	80	50	30
OxFord flowers 102	102	40 to 258	20 to 200	20 to 58
Caltech/UCSD birds	200	6033	4000	2033
Caltech 101 airplanes	101	40 to 800	20 to 600	20 to 200

**Table 3:** The initial parameters of algorithms.

Algorithm	Parameter	Value
SFL	Maximum permitted change in a frog's location	10
	Number of memeplex	20
	Number of frogs	30

ACO	Pheromone update constant (*Q*)	15
	Global pheromone decay rate (*pg*)	0.7
	Visibility sensitivity (*β*)	7
	Population size	70
	Number of ants	15
	Maximum number of iterations	35
	Local pheromone decay rate (*pt*)	0.6
	Initial pheromone (*τ*)	1e-06
	Pheromone sensitivity (*α*)	1
	Pheromone constant (*q*)	1

BFSO	Probability of elimination	0.1
	Spreading percentage %*σ*	0.4
	Population size	60
	Number of bacteria	20
	Maximum number of iterations	35

WHO	Strategies	Decreasing the value of *a*
	Whales attacking	Encircling
	Max a	5
	Probability of choosing spiral model	*P* ∈ [0, 1]
	Probability of choosing shrinking encircling	*p* ∈ [0, 1]
	Population size	70
	Number of whales	15
	Maximum number of iterations	35

**Table 4:** Experimental results for the oxford flowers 17 dataset.

Technique	MSE (AVE ± STD)	Classification rate (%)	Training time
LeNet 5	0.190425 ± 0.031687	88	14 minutes
ACO-LeNet 5	0.121689 ± 0.011574	90	16 minutes
BFSO-LeNet 5	0.085050 ± 0.034945	91	25 minutes
WO-LeNet 5	0.032228 ± 0.039778	94	18 minutes
SFLA-LeNet 5	0.009210 ± .039100	97	23 minutes

**Table 5:** Experimental results for the oxFord flowers 102 dataset.

Technique	MSE (AVE ± STD)	Classification rate (%)	Training time
LeNet 5	0.040320 ± 0.002470	90	51 minutes
ACO-LeNet 5	0.024881 ± 0.002472	95	58 minutes
BFSO-LeNet 5	0.008026 ± 0.007900	93	67 minutes
WO-LeNet 5	0.0229 ± 0.0032	91	64 minutes
SFLA-LeNet 5	0.003026 ± 0.001500	97	65 minutes

**Table 6:** Experimental results for the Caltech/UCSD birds dataset.

Technique	MSE (AVE ± STD)	Classification rate (%)	Training time
LeNet 5	0.0321 ± 0.0045	92	97 minutes
ACO-LeNet 5	0.0019 ± 8.4257*e*−04	97	101 minutes
BFSO-LeNet 5	0.0078 ± 8.2189*e*−02	93	109 minutes
WO-LeNet 5	0.0045 ± 8.7654*e*−03	96	103 minutes
SFLA-LeNet 5	0.0021 ± 9.4298*e*−05	98	105 minutes

**Table 7:** Experimental results for the Caltech 101 airplanes dataset.

Technique	MSE (AVE ± STD)	Classification rate (%)	Training time
LeNet 5	0.050420 ± 0.003170	92	49 minutes
ACO-LeNet 5	0.031841 ± 0.004123	94	52 minutes
BFSO-LeNet 5	0.072218 ± 0.079235	93	57 minutes
WO-LeNet 5	0.00319 ± 0.0042	96	53 minutes
SFLA-LeNet 5	0.00286 ± 0.009700	97	55 minutes

## Data Availability

These datasets are public datasets and are available at the following links: https://www.robots.ox.ac.uk/~vgg/data/flowers/17/http://www.vision.caltech.edu/Image_Datasets/Caltech101/http://www.vision.caltech.edu/visipedia/CUB-200.htmlhttps://www.robots.ox.ac.uk/~vgg/data/flowers/102/.
